The article "Regulatory Networks of Prognostic mRNAs in Pediatric Acute Myeloid Leukemia" was retracted in 2022. Reason: concerns about the peer review.

# Regulatory Networks of Prognostic mRNAs in Pediatric Acute Myeloid Leukemia

**DOI:** 10.1155/2022/2691997

**Published:** 2022-01-05

**Authors:** Hao Zhang, Liqin Cheng, Cong Liu

**Affiliations:** ^1^Beijing Shijitan Hospital Affiliated to Capital University of Medical Sciences, Neonatology, No. 10 Tieyi Road, Yanggang Store, Haidian District, Beijing 100038, China; ^2^Beijing Space Center Hospital Paediatrics, 15 Yuquan Road, Haidian District, Beijing 100049, China; ^3^Beijing New Century Women and Children Hospital Paediatrics, 15 Wangjing North Road, Chaoyang District, Beijing 100102, China

## Abstract

Acute myeloid leukemia (AML) in children refers to a malignant tumor caused by the abnormal proliferation of immature myeloid cells in the bone marrow and peripheral blood. The prognosis of patients with pediatric acute myeloid leukemia (AML) remains poor, highlighting the need for improved targeted therapy. The expression data of lncRNAs, mRNAs, and miRNAs and survival information of pediatric AML patients were collected from The Cancer Genome Atlas (TCGA) database. Cox regression analysis was used to screen the lncRNAs, mRNAs, and miRNAs that significantly affect the overall survival (OS) of patients as OS-related genes (included lncRNAs, mRNAs, and miRNAs). Enrichment analysis and protein-protein interaction (PPI) network construction were performed for the OS-related mRNAs. We further established a ceRNAs regulatory network. In addition, the potential prognostic role of genes was further evaluated by risk score. We have identified 5275 lncRNAs, 176 miRNAs, and 6221 mRNAs that significantly affect the prognosis of pediatric AML patients. It is worth noting that OS-related mRNAs are mainly involved in ribosome, RNA transport, and spliceosome. We identified the top 10 most connected mRNAs in the PPI network as important mRNAs and constructed a ceRNAs regulatory network (including NCBP2, RPLP0, UBC, RPS2, and RPS9). The risk score and nomogram results suggest that NCBP2 may be a risk factor for pediatric AML, while RPLP0, UBC, RPS2, and RPS9 may be protective factors. Our results construct 5 gene signals as new prognostic indicators for predicting the survival of pediatric AML patients. Our research has demonstrated the ceRNAs regulatory network may become a new target for pediatric AML treatment.

## 1. Introduction

AML is one of the more common types of childhood acute leukemia [1]. The pathogenesis of AML is characterized by the increased self-renewal ability of leukemia cells and the obstruction of apoptosis, which leads to a large number of proliferation and accumulation in the bone marrow and other hematopoietic tissues, which inhibits normal hematopoietic function [2]. Moreover, leukemia cells are highly aggressive and infiltrate other tissues and organs, causing varying degrees of anemia, infection, fever, hemorrhage, and swelling of the liver, spleen, and lymph nodes. According to global statistics, the proportion of AML in childhood acute leukemia is about 20%, and the cure rate is close to 70% [1]. In the US, the incidence of AML is about 18% of all childhood leukemias, and the incidence has been on the rise. The fatality rate accounts for about half of all childhood leukemias [3]. It is estimated that 8.5 out of every million children will have acute myeloid leukemia [4]. With the improvement of the modern medical technology, the treatment plan for AML is constantly updated, coupled with the successive research and development of new drugs. The survival rate of AML has been greatly improved, and the survival time of children has been prolonged. Studies have shown that the survival rate for AML in eastern European countries has risen from 31% to 63%, and the 5-year overall survival rate has risen from 41% to 71% [5]. In the Netherlands, AML rose from 40% in early 1990 to 74% in 2010–2015. Despite this, the recurrent episodes and high mortality of AML still plague countless families and patients [6]. Identifying an effective diagnosis of AML and providing a therapeutic target has also become a problem that needs to be solved in the world.

The miRNA and lcRNA are a large number of functional noncoding RNAs in the body, which can regulate transcription. The miRNA and lcRNA have specific structures and biological functions and participate in various physiological and pathological processes of the body [7–12]. At present, studies have shown that the role of the lncRNA and miRNA in tumors has been initially recognized, and some studies have shown that the lncRNA and miRNA can be used as biomarkers of AML [13, 14]. So far, no diagnostic targets with strong specificity and sensitivity for AML have been identified. The ceRNA network detection method for the lncRNA and miRNA may bring new enlightenment to the prognosis monitoring and treatment of AML.

With the popularization of genetic detecting, many new detection methods related to AML have emerged, and genomics-based methods have been promoted to monitor treatment response and adjust programs to improve treatment efficacy and prolong survival [1]. However, so far, the mechanism of the occurrence and development of AML is still unclear. The analysis of differential genes after the occurrence of the disease is of great significance to the prognostic diagnosis and treatment of AML. However, due to the limitation of technical conditions, the advantage of the targeting for accurate disease judgment cannot be brought into play. Therefore, it is very likely that there are some new genes related to the prognosis of AML. In this study, the previous AML gene expression data was reanalyzed to screen potential new targets for the prognostic diagnosis and treatment of AML.

## 2. Materials and Methods

### 2.1. Data Collection and Processing

Gene expression profiles and survival information were collected from The Cancer Genome Atlas (TCGA) database. The miRNA expression profiles were based on 366 pediatric AML samples, and the lncRNA and mRNA expression profiles were based on 187 pediatric AML samples.

Cox regression analysis was used to identify genes (miRNAs, lncRNAs, and mRNAs) influencing the overall survival (OS) of pediatric AML patients and considered as OS-related genes. A *P* value <0.05 was considered significant.

### 2.2. Biological Function Analysis

The Gene ontology (GO) and Kyoto encyclopedia of genes and genomes (KEGG) pathway enrichment analysis of OS-related mRNAs were analyzed using Enrichr R package. A *P* value <0.05 were used as the cutoff criteria. GO results included biological processes (BP), cellular components (CC), and molecular functions (MF).

### 2.3. Construction of the Regulated Network

The target-regulated lncRNAs of OS-related miRNAs were predicted by using miRandaonline tool. The target-regulated mRNAs of OS-related miRNAs were predicted by using miRTarBase online tool. The protein-protein interaction (PPI) network of OS-related mRNAs was constructed, and the top 10 degrees of connectivity in the network was screened as important mRNAs. Subsequently, the target lncRNAs and mRNAs were comparatively analyzed with OS-related lncRNAs and important mRNAs. The ceRNAs regulatory networks of important mRNAs were finally constructed. RPLP0 is a ribosomal protein, and it has a regulatory effect on protein synthesis and cell cycle [15]. In addition, RPLP0 is associated with a variety of tumors. RPLP0 is highly expressed in the tumor group through the detection of endometrial cancer and ovarian cancer patients and showed that RPLP0 is closely related to human tumors and may become a prognostic marker of gynecological diseases [16]. Studies have shown that RPLP0 interacts with cathepsin *X*/*Z* to regulate the inactivation of the apoptosis signaling pathway in gastric cancer cells [17]. Moreover, the low expression of RPLP0 in gastric cancer cells can lead to gastric cancer cell cycle arrest. In the related research of AML, RPLP0 is highly expressed in AML [18]. Our research shows that RPLP0 may be closely related to the prognosis of AML. Moreover, RPLP0 is beneficial to the overall survival of AML patients.

### 2.4. Survival Analysis and Risk Regression Analysis

Kaplan–Meier (K–M) estimator was performed using the survival R package. Cox regression analysis for OS-related mRNAs in the TCGA dataset was performed. According to the median value of the risk score calculated by the Cox regression coefficient, patients were divided into high-risk groups and low-risk groups. The area under the receiver operating characteristic curve (AUC) value was calculated.

## 3. Results

### 3.1. Prognosis-Associated Genes in Pediatric AML

In order to identify the genes that affect the prognosis of children with AML, we collected the expression data of lncRNAs, miRNAs, and mRNAs from the TCGA database. Using Cox regression analysis, 5275 lncRNAs, 176 miRNAs, and 6221 mRNAs that significantly affect the prognosis of patients were identified (Figures 1(a)–1(c)).

### 3.2. Enrichment Analysis of OS-Related mRNAs

In order to explore the molecular dysregulation mechanism of prognostic-related mRNAs in AML, we conducted a biological function enrichment analysis. The results for biological processes (BPs) showed that protein targeting to ER, ncRNA processing, and cotranslational protein targeting to membrane were enriched (Figure 2(a)). For cellular component (CC), nucleus, nuclear lumen, and intracellular membrane-bounded organelle were significantly enriched (Figure 2(b)). Then, RNA binding, mRNA binding, and 3′-5′ exonuclease activity were enriched for the molecular function (MF) (Figure 2(c)). Additionally, KEGG signaling pathway terms were also significantly enriched, which mainly involved ribosome, RNA transport, and spliceosome (Figure 2(d)).

### 3.3. Construction of ceRNAs Regulated Networks

Through the Miranda online prediction website, we have identified lncRNAs targeted by OS-related miRNAs. By comparing with OS-related lncRNAs, we identified 94 OS-related target lncRNAs (Figure 3(a)). Using the miRTarBase online prediction website, 6054 target mRNAs of OS-related miRNAs were predicted and compared with OS-related mRNAs, 437 targeted and regulated OS-related mRNAs were obtained (Figure 3(b)). Furthermore, by constructing the PPI network of OS-related mRNAs, we screened the top 10 mRNAs with the highest degree of connection in the network as important mRNAs (Figure 3(c)). Finally, we constructed the lncRNA-miRNA-mRNA ceRNAs network of important mRNAs (Figure 3(d)). NCBP2, RPLP0, UBC, RPS2, and RPS9 of important mRNAs were found in the network and considered as candidate genes. By constructing a ceRNAs network that affects the prognosis of AML patients, we have identified 5 candidate genes. NCBP2 is a 20 kDa gene located at 3q29 [19], which is mainly involved in the splicing process of precursor mRNA [20]. Currently, studies have shown that the expression of NCBP1 in tumor tissues is significantly increased. In subsequent studies, it was reported that NCBP2 may be a regulatory gene of miR-193a-5p [21]. This also further illustrates the role of NCBP2 in tumors. In this study, NCBP2 may be a genetic risk factor for AML patients, which indicates that NCBP2 can be used as a potential prognostic target for AML.

### 3.4. Candidate Genes Affect the Prognosis of Pediatric AML Patients

The risk scores were calculated for 5 candidate genes, and the median risk score was used to divide AML patients into high-risk groups and low-risk groups. In the TCGA dataset, NCBP2 was highly expressed in the high-risk group, and RPLPO, UBC, RPS2, and RPS9 were upregulated in the low-risk group (Figure 4(a)). The median risk score predicts AUC ≥0.7 for 1-, 3-, and 5-year survival rates in AML patients (Figure 4(b)). Compared with the low-risk score, it has a high-risk score (Figure 4(c)).

Moreover, we constructed a nomogram of candidate genes. RPLP0 and UBC are beneficial to the overall survival rate of AML patients, and NCBP2 may be a genetic risk factor for AML patients (Figure 5(a)). The calibration chart was used for verification to evaluate the accuracy of the alignment model, and the accuracy was good (Figure 5(b)). In addition, the KM curve shows the bone marrow of AML patients with high expression of NCBP2 and low expression of RPLP0, UBC, RPS2, and RPS9 (Figure 5(c)).

## 4. Discussion

In this study, 11672 genes related to the prognosis of AML were identified from the TCGA database. Further analysis showed that NCBP2, RPLP0, UBC, RPS2, and RPS9 can be used as prognostic diagnostic markers for AML. Moreover, in the high-risk group, NCBP2 expression was significant. Significant expression of RPLP0, UBC, RPS2, and RPS9 in the low-risk group. Moreover, RPLP0 and UBC are beneficial to the overall survival rate of AML patients, and NCBP2 may be a risk factor for AML patients.

AML is highly heterogeneous. Therefore, it is of great significance to seek indicators for judging the prognosis and to guide the design of individualized treatment plans. The currently identified prognostic factors affecting AML mainly include the age, peripheral blood leukocyte count, secondary leukemia, and karyotype [22]. Among them, the karyotype is of great value to prognostic judgment, and there are obviously different treatment responses in patients with the same or normal karyotype immediately [23]. Genetic detecting can not only effectively warn the occurrence and diagnosis of diseases, but also provide targeted therapeutic targets for clinical treatment [24]. In this study, through the analysis of gene expression and the overall survival of patients, we found as many as 11672 prognostic-related genes in AML patients. Research on these genes can improve disease monitoring and treatment options for AML.

UBC is a highly conserved polypeptide that participates in a variety of signal transduction and life processes. Studies have shown that UBC participates in the process of heat stress response, is the main provider of ubiquitin factors in heat stress response, and maintains the stress response and heat tolerance of cells [25]. In addition, UBC-deficient mice can cause embryonic mouse death and affect liver development [26]. Moreover, UBC is also a diagnostic biomarker for breast cancer [27]. In this study, the expression of UBC was significantly upregulated and has a high research value for AML.

Both RPS2 and RPS9 are ribosomal proteins and are involved in ribosome formation and protein synthesis [28]. The current research shows that RPS2 has been reported in a lot of tumor-related research [29–34]. Moreover, RPS2 has been reported as a new target for the treatment of prostate cancer [30]. RPS9 may serve as a biomarker for lung squamous cell carcinoma [35].

## 5. Conclusion

In summary, our results indicate that NCBP2, RPLP0, UBC, RPS2, and RPS9 are closely related to the prognosis of AML and may be potential therapeutic targets for AML. However, the role of RPS2 and RPS9 in AML has not yet been reported. In this study, RPS2 and RPS9 are closely related to the prognosis of AML and have great potential to be developed in the prognostic diagnosis of AML and the application of drug treatment targets.

## Figures and Tables

**Figure 1:** Identification of genes influencing pediatric AML patient prognosis. (a) Volcano plot of OS-related lncRNAs in the TCGA dataset. (b) Volcano plot of OS-related miRNAs in the TCGA dataset. (c) Volcano plot of OS-related mRNAs in the TCGA dataset. Red indicates high risk with the coeffiecient of Cox regression >0, and blue indicates low risk with the coefficient of Cox regression <0.

**Figure 2:** Enrichment of GO and KEGG pathways for OS-related mRNAs in AML. (a) The top 10 significant biological processes for OS-related mRNAs. (b) The top 10 significant cellular components for OS-related mRNAs. (c) The top 10 significant molecular functions for OS-related mRNAs. (d) Significant enriched KEGG pathways for OS-related mRNAs.

**Figure 3:** Identification of the regulated networks in AML. (a). Intersection of targeted lncRNAs of OS-related miRNAs and OS-related lncRNAs. (b) Intersection between targeted mRNAs of OS-related miRNAs and OS-related mRNAs. (c) The top ten degree of connectivity in the PPI network for OS-related mRNAs. The redder the color, the higher the degree of connectivity. (d) The network of important mRNAs with miRNAs and lncRNAs. Red is mRNAs, orange is miRNAs, and blue is lncRNAs.

**Figure 4:** Cox risk score of candidate genes influences AML patient prognosis in the TCGA dataset. (a) Distribution of candidate mRNAs‐based risk scores, mRNAs expression levels, and patient survival durations in the TCGA dataset. (b) AUC values for the risk median score to predict 1-year, 3-year, and 5-year survival of AML patients. (c) Kaplan–Meier curves of OS for AML patients based on the risk score in the TCGA dataset.

**Figure 5:** Evaluation of candidate genes. (a) The nomogram model constructed with expression of candidate genes to predict the prognosis of AML patients. (b) The calibration curves for the nomogram model. (c) Kaplan–Meier curves of candidate genes for OS of AML patients.

## Data Availability

The datasets used and/or analyzed during the current study are available from the corresponding author on reasonable request.
